# Urinary Matrix Metalloproteinase-9 and Nephrin in Idiopathic Membranous Nephropathy: A Cross-Sectional Study

**DOI:** 10.1155/2021/1620545

**Published:** 2021-10-18

**Authors:** Akankwasa Gilbert, An Changjuan, Cheng Guixue, Liu Jianhua, Qin Xiaosong

**Affiliations:** Department of Clinical Laboratory, Shengjing Hospital of China Medical University, No. 36, Sanhao Street, Heping District, Shenyang, Liaoning Province 110004, China

## Abstract

**Aim:**

Idiopathic membranous nephropathy (IMN) has a varied clinical course that requires accurate prediction as a prerequisite for treatment administration. Currently, its prognosis relies on proteinuria, a clinical parameter whose onset lags behind kidney injury. Increased urinary excretion of matrix metalloproteinase-9 (MMP-9) and nephrin has been reported in a number of IMN-like glomerular diseases in which they reflected disease severity. However, little or nothing is known of the importance of these biomarkers in IMN, a major cause of adult nephrotic syndrome. To highlight their potential, we measured both biomarkers and assessed their relationships with key parameters of renal function in IMN.

**Methods:**

We quantified urinary MMP-9 and nephrin in 107 biopsy-proven IMN patients and 70 healthy subjects by enzyme-linked immunosorbent assay (ELISA). We then compared biomarker levels between patients and healthy subjects and among patients with different clinical features. We also determined the relationship of each biomarker with proteinuria and the estimated glomerular filtration rate (eGFR).

**Results:**

Urinary MMP-9 and nephrin were significantly higher in IMN compared to healthy controls. Unlike nephrin, MMP-9 correlated significantly with proteinuria and was significantly higher among patients with nephrotic range proteinuria. Both biomarkers were correlated with eGFR, but only MMP-9 was significantly higher in patients with eGFR less than 90 ml/min/1.73 m^2^.

**Conclusion:**

Our findings suggest that urinary MMP-9 holds a greater potential than urinary nephrin in monitoring the severity of IMN.

## 1. Introduction

Regarded as a single organ autoimmune disorder, idiopathic membranous nephropathy (IMN) is a subtype of membranous nephropathy to which many cases of adult nephrotic syndrome are attributed. IMN affects more men than women, and its prevalence among the primary glomerular diseases is on an increasing trend [1, 2]. The pathogenesis of IMN involves destruction of the glomerular basement membrane by an immune-mediated process that results into massive proteinuria. This process is facilitated by either phospholipase A_2_ receptors (PLA_2_R), the major glomerular antigen, or the other minor antigens such as thrombospondin type 1 domain-containing 7A (THSD7A) [3]. Present in about 80% of cases, the serum PLA_2_R antibodies are among the few candidate markers for the prognosis of IMN [4, 5].

Presently, there is a scarcity of biomarkers capable of predicting the course of IMN, especially in its early stages. Proteinuria is the only prognostic parameter recommended by the 2012 kidney disease improving global outcomes (KDIGO) clinical practice guidelines. However, the use of proteinuria to predict the course of IMN is not without challenges. While proteinuria in the subnephrotic range (defined as urine protein < 350 mg/mmolCr) was found associated with a reduced risk of end-stage renal disease (ESRD) and could predict excellent long-term survival of kidneys [6, 7], it occurs after significant renal damage. Moreover, it takes a urine protein level as high as 2.43 g/day at baseline to predict which patient will suffer a severe form of IMN within a year [7]. Accordingly, a search for alternative biomarkers capable of predicting the course of IMN before significant renal damage is warranted.

Matrix metalloproteinase-9 (also known as gelatinase B) and nephrin are some of the early markers of glomerular dysfunction. The urinary excretion and activity of these markers are already known to reflect the severity of nephrotic syndrome other glomerular diseases [8–13]. Derived from glomerular podocytes, nephrin and MMP-9 influence glomerular functions; MMP-9 degrades type IV collagen of the glomerular basement membrane [14, 15] while nephrin checks proteinuria and facilitates podocyte recovery after injury [16].

The potential utility of these biomarkers has been documented in a number of glomerular diseases including diabetic nephropathy, Henoch-Schonleinpurpura, minimal change disease, and focal segmental glomerulosclerosis [8, 11–13]. However, no attempt has been made at assessing their potential utility in IMN. Thus far, nephrin and MMP-9 have been studied in only disease models with important revelations such as enhanced glomerular expression of MMP-9 and dissociation of nephrin from podocin prior to the onset of proteinuria [17, 18].

Despite these findings, the diagnostic and prognostic potential of these biomarkers has never been studied in human subjects. Only MMP-9 has had its diagnostic and prognostic potentials studied but in only childhood forms nephrotic syndrome [8, 9, 12]. As such, it remains to be determined if urinary nephrin and MMP-9, as individual markers or in combination with other biomarkers, could be important in an adult form of nephrotic syndrome such as IMN. The purpose of this is study therefore is to quantify urinary MMP-9 and nephrin, assess their relationship with parameter renal function, and deduce their importance in the management of IMN.

## 2. Materials and Methods

### 2.1. Ethical Approval

The study was approved by the research ethics committee of Shengjing Hospital of China Medical University.

### 2.2. Recruitment of Idiopathic Membranous Nephropathy Patients

107 biopsy-proven IMN patients were recruited from the hospital's nephrology department from March 2018 to January 2020. At the time of recruitment, none of the patients had received IMN treatment. Participants were screened for all possible causes of secondary membranous nephropathy and other kidney diseases. Those found with neoplasms, cancers, diabetes, autoimmune diseases such as systemic lupus erythematosus, purpura nephritis, infections such as hepatitis B and hepatitis C viruses, and other comorbidities were excluded. Furthermore, patients were also excluded on the basis of history of exposure to drugs and chemicals such as rifampicin, captopril, probenecid, ibuprofen, birth control pills, diclofenac, formaldehyde, and volatile hydrocarbons. Renal biopsies were taken and subjected to an examination by light microscopy, electron microscopy, and fluorescence microscopy.

### 2.3. Recruitment of Healthy Controls

Healthy controls were recruited from the health examination centre of Shengjing Hospital of China Medical University. Those found with urinary tract infections or any other abnormalities were excluded.

### 2.4. Sample Collection and Storage

Urine and blood samples were collected from participants before renal biopsies. Blood was collected into plain vacutainers and allowed to clot thoroughly before centrifuging to obtain serum while random urine samples were collected using clean plastic containers and centrifuged at 1000g for 20 minutes to obtain the supernatants. Both sera and urine supernatants were kept at -80°C pending analysis.

### 2.5. Data Collection

#### 2.5.1. Basic Clinical and Demographic Characteristics

Demographic and clinical information about the recruited participants was collected from the hospital's Laboratory Information System (LIS) and Health Information System (HIS). The assay of biochemical parameters such as urine protein, serum creatinine, serum urea, serum cystatin C (Cys-C), blood glucose, total serum protein, serum albumin, and urine creatinine (UCr) was carried out using an ARCHITECT C 16000 biochemical analyzer (Abbott, USA). The estimated glomerular filtration rate (eGFR) was calculated using the chronic kidney disease epidemiology collaboration (CKD-EPI) formula: eGFR = 141 × (serum Cr/*K*) *a* × (0.993) age × 1.018 (*K* value: female = 0.7, male = 0.9; *a* value: female, serum Cr ≤ 0.7, *a* = −0.329, serum Cr > 0.7, *a* = −1.209; *a* value: male, serum Cr ≤ 0.9, *a* = −0.411, serum Cr > 0.9, *a* = −1.209).

#### 2.5.2. The Assay of Urinary Nephrin and Matrix Metalloproteinase-9

The levels of urinary nephrin and MMP-9 were determined in accordance with instructions as laid down in the operator's manual kits (http://www.cloud-clone.com/manual/ELISA-Kit-for-Matrix-Metalloproteinase-9-(MMP9)-SEA553Hu.pdf and http://www.cloud-clone.com/manual/ELISA-Kit-for-Nephrin-(NPHN)-SEA937Hu.pdf). The concentrations of nephrin and MMP-9 were obtained, standardized with urine creatinine, and reported.

### 2.6. Criteria for Assessing Associations of Urinary Nephrin and Matrix Metalloproteinase-9 with Parameters of Renal Function in Idiopathic Membranous Nephropathy

Urinary nephrin and MMP-9 were assessed for possible associations with urinary protein and eGFR as follows:

#### 2.6.1. Association of Urinary Nephrin and Matrix Metalloproteinase-9 with Proteinuria

To determine the association of urinary nephrin and MMP-9 with proteinuria, we first established the correlation of each biomarker with proteinuria in all patients. We then grouped patients into two groups, i.e., the subnephrotic range group (proteinuria < 350 mg/mmolCr) and the nephrotic range group (proteinuria > 350 mg/mmolCr), and compared their levels.

#### 2.6.2. Association of Urinary Nephrin and Matrix Metalloproteinase-9 with Estimated Glomerular Filtration Rate

To assess the associations of urinary nephrin and MMP-9 with renal function, we first determined the correlation of eGFR with each biomarker. We then stratified patients into two groups (i.e., patients with eGFR less than 90 ml/min/1.73 m^2^ and those with eGFR greater than 90 ml/min/1.73 m^2^) and compared the biomarker levels.

### 2.7. Statistical Analysis

The data was analyzed using SPSS version 19. The normality of data was tested with the Kolmogorov–Smirnov test. Variables with normal distributions were presented as mean ± standard deviation while those with skewed distribution were presented as median (interquartile range). Sex ratio was compared using the chi-square test while group means and medians were compared using independent samples *t*-test and Mann-Whitney *U* test as appropriate. The correlations were determined with Spearman's and Pearson's correlations where applicable. All tests were two-sided, and *P* values less than 0.050 were considered significant.

## 3. Results

### 3.1. Comparison of Demographic and Basic Clinical Characteristics between Patients and Healthy Controls

Information regarding demographic and basic clinical characteristics of study participants is as summarized in Table 1.

There was no significant difference in age, sex ratio, fasting blood sugar, creatinine, and eGFR between patients and healthy subjects. However, there was significant difference in levels of serum albumin, serum total protein, serum cystatin C, serum urea, diastolic blood pressure, systolic blood pressure, and urine protein.

### 3.2. Comparison of Urinary Nephrin and Matrix Metalloproteinase-9 between Patients and Healthy Controls

Urinary nephrin and MMP-9 were significantly increased in IMN patients compared to the healthy subjects (Table 2).

Unlike MMP-9 that was detectable in both patients and healthy controls, nephrin was detectable only among patients.

### 3.3. Comparison of Urinary Levels of Nephrin and Matrix Metalloproteinase-9 between Patients with and without Nephrotic Syndrome

As shown in Table 3, the urinary levels of both biomarkers were higher among patients with nephrotic syndrome compared to those without.

Urinary MMP-9 was significantly increased in patients with nephrotic range proteinuria compared to patients with subnephrotic range proteinuria. Unlike urinary MMP-9 however, the increase in urinary nephrin did not reach statistical significance.

### 3.4. Comparison of Urine Biomarker Levels between Patients with Estimated Glomerular Filtration Rate below and above 90 ml/min/1.73m^2^

To establish whether the urine excretion of nephrin and MMP-9 varies between patients with differences in renal function, we compared the biomarker levels between patients with eGFR less than 90 ml/min/1.73 m^2^ and those with eGFR greater than 90 ml/min/1.73 m^2^. As shown in Table 3, only urinary MMP-9 was significantly increased among patients with eGFR less than 90 ml/min/1.73 m^2^. There was no significant difference in the levels of urinary nephrin between the two groups.

### 3.5. Assessment of Linearity between Urine Biomarkers and Established Parameters of Renal Function

To assess whether urinary levels of nephrin and MMP-9 are related with major parameters of renal function, we determined the correlation of each biomarker with eGFR and proteinuria. As shown in Table 4, urinary MMP-9 was significantly correlated with proteinuria and eGFR while urinary nephrin was significantly correlated with only eGFR.

## 4. Discussions

The management of IMN is still problematic due to lack of reliable biomarkers capable of predicting patient outcomes in the early stages. For so long, the prediction of patient outcomes has relied on proteinuria, a clinical parameter whose onset lags behind kidney damage. In this study, we examined the association of urinary nephrin and MMP-9 with key parameters of renal function with an aim of deducing their potential roles in the management of IMN.

The levels of nephrin and MMP-9 were significantly increased among patients compared to the healthy controls (Tables 3 and 4). Unlike MMP-9 however, nephrin was undetectable in the healthy subjects. This observation is consistent with studies by Bienias and Sikora [12] and Musial et al. [8] which reported higher levels of MMP-9 in other forms of glomerular kidney diseases. Our results are also consistent with those of Wang et al. [10] in which urinary nephrin was detectable only in patients but not healthy controls. The levels of the two biomarkers reflect renal abnormalities among IMN patients. Indeed, these findings compliment and render credence to studies in Heymann nephritis (a disease model of IMN) in which MMP-9 was upregulated and nephrin dissociated from glomerular podocytes [17, 18].

In the current study, urinary MMP-9 in patients with nephrotic syndrome was not only higher but also correlated with proteinuria (Tables 3 and 4), an observation consistent with the findings in Henoch-Schonleinpurpura [9]. However, this was not the case with nephrin whose level in subjects with nephrotic syndrome was neither significantly high nor correlated with proteinuria.

Both biomarkers were significantly correlated with eGFR (Table 4), but only MMP-9 was significantly higher among patients with eGFR less than 90 ml/min/1.73m^2^ (Table 3). The eGFR is a general parameter used to determine the rate of renal function decline [19] and to predict the occurrence of ESRD in chronic kidney disease (CKD) [20]. By virtue of its correlation with eGFR and increased levels among patients with eGFR less than 90 ml/min/1.73m^2^, our findings suggest that urinary MMP-9 holds a greater potential as a surrogate marker of renal function.

Our findings suggest that MMP-9 is superior to nephrin at reflecting decline in renal function. Presently, there is scanty literature regarding the ability of urinary nephrin and MMP-9 to reflect renal function, especially in CKD. However, it seems that urinary nephrin is only a qualitative marker of glomerular damage occurring in the early stages of IMN and may carry no prognostic value. To the extent that urinary nephrin was detectable in patients with eGFR greater than 90 ml/min/1.73 m^2^ (Table 3) and not in the healthy subjects (Table 2), the results of this study are in support of this opinion. Also, the lack of significant correlation with proteinuria as observed in the current study further supports the idea that urinary nephrin is incapable of reflecting disease activity.

Regarding the suitability of urinary MMP-9 as a biomarker reflecting the decline in renal function, our results are in harmony with the previous studies which reported significant urinary levels that correlated well with eGFR [20, 21]. In addition to degrading the GBM, MMP-9 also promotes abnormal mesangial proliferative changes [22]. MMP-9 initiates fibrosis, a process that irreversibly compromises glomerular functions. By cleaving osteopontin, a macrophage chemoattractant, MMP-9 activates transforming growth factor-*β* (TGF-*β*), a cytokine that induces renal fibrosis [23, 24].

IMN is a primary glomerular disease whose severity is dependent on the extent of glomerular damage. The glomerular podocytes are targeted for immune destruction by the anti-PLA_2_R. Depending on the magnitude of the insult, the injured podocytes can undergo apoptosis or a series of adaptational changes. The adaptational changes of podocytes include rearrangement of their actin cytoskeleton, a process that leads to foot process effacement and detachment of expressed proteins such as nephrin [25]. As the glomerular insult rages on, more and more apoptotic podocytes detach and wash down the urinary space causing a proportionate increase in total proteinuria and the podocyte-expressed proteins. This explains why urinary nephrin was higher (though not significantly) among patients with nephrotic range proteinuria compared to those with nephrotic range proteinuria (Table 3).

MMP-9 belongs to the gelatinase family. Gelatinases are a group of enzymes that cleave type IV collagen which is a major constituent of the GBM. Although the potential of MMP-9 to reflect the severity of IMN has not been studied, MMP-9 is a recognized player in the pathogenesis of several glomerular diseases [22]. The exposure of the glomerular podocytes to albumin enhanced the activity and glomerular expression of MMP-9 [26, 27], a phenomenon that could be true for IMN. Therefore, we speculate that following the immune-mediated kidney injury in IMN, increased permeability of serum proteins exposes podocytes to albumin upregulating MMP-9's expression and its consequent urinary shedding. This, perhaps, explains the positive relationship observed between MMP-9 and proteinuria in the present study.

Identification of MMP-9 as a potential marker for the severity of IMN is of utmost importance to its management. IMN has a variable clinical course with one-third of the patients progressing to ESRD. Such a progression can be prevented or reduced if its severity and prognosis are accurately determined and appropriate treatments administered in time.

## 5. Conclusion

The current study has for the first time demonstrated that a relationship exists between urinary MMP-9 and the renal parameters in IMN. Unlike nephrin, MMP-9 exhibited significant association with proteinuria, a parameter currently used to assess the severity of IMN. Accordingly, MMP-9 holds a greater potential in monitoring the severity of IMN. To further elucidate MMP-9's potential, more studies are needed especially in determining its relationship with the IMN-specific markers such as PLA_2_R antibodies.

The limitations of this study include the design which did not permit assessment of biomarker levels over time and the lack of information regarding the other IMN-specific antibodies which hold pathogenic and prognostic roles. Future studies should investigate the urine excretion patterns of MMP-9 in a prospective manner for better appreciation of its prognostic potential for IMN.

## Figures and Tables

**Table 1:** Comparison of demographic and basic clinical characteristics between patients and healthy controls.

Parameters	Healthy controls (*n* = 70)	IMN patients (*n* = 107)	*P* value
Sex (male/female)	45/25	67/40	0.475
Age (years)	46.78 ± 5.81	48.57 ± 12.86	0.277
Diastolic blood pressure (mm/Hg)	77.00 (67.00-87.00)	80.00 (70.00-90.00)	0.020
Systolic blood pressure (mm/Hg)	121.00 (113.00-133.00)	123.00 (123.00-133.00)	0.035
Fasting blood glucose (mmol/l)	4.37 ± 0.49	4.45 ± 0.57	0.379
Serum protein(g/l)	74.35 (71.60-76.55)	46.20 (38.10-52.60)	0.015
Serum albumin (g/l)	47.20 (45.27-48.62)	25.40 (19.60-33.00)	0.041
Urine protein (mg/*μ*mol Cr)	3.26 (1.93-4.91)	372.18 (181.12-734.65)	0.021
Serum cystatin C (mg/l)	0.82 ± 0.13	1.24 ± 0.32	0.011
Serum creatinine (*μ*mol/l)	66.43 ± 16.40	68.78 ± 17.37	0.370
Serum uric acid (*μ*mol/l)	313.66 ± 56.45	348.78 ± 69.52	0.023
Serum urea (mmol/l)	4.97 ± 1.35	5.92 ± 1.76	0.033
eGFR (ml/min/m^2^)	104.60 (90.25-118.69)	104.82 (96.76-112.20)	0.798

IMN: idiopathic membranous nephropathy; eGFR: estimated glomerular filtration rate.

**Table 2:** Comparison of urinary levels of nephrin and matrix metalloproteinase-9 in healthy and idiopathic membranous nephropathy.

Biomarkers	Healthy controls (*n* = 70)	IMN patients (*n* = 107)	*P* value
Urinary MMP-9 (ng/*μ*molUCr)	0.31 (0.21-0.46)	0.61 (0.26-1.87)	0.002
Urinary nephrin (ng/*μ*molUCr)	Undetectable.	0.60 (0.23-1.02)	N/A

UCr: urine creatinine; IMN: idiopathic membranous nephropathy; MMP-9: matrix metalloproteinase-9; N/A: not applicable.

**Table 3:** Urinary levels of MMP-9 and nephrin in patients with different clinical features of idiopathic membranous nephropathy.

Biomarkers (ng/*μ*molUCr)	Level of proteinuria (mg/mmolCr)			eGFR (ml/min/1.73 m^2^)		
	<350 (*n* = 65)	>350 (*n* = 42)	*P* value	>90 (*n* = 86)	<90 (*n* = 21)	*P* value
MMP-9	0.40 0.21-0.85	1.11 0.58-2.74	0.014	0.50 0.21-1.23	2.02 0.51-3.62	0.020
Nephrin	0.66 ± 0.58	0.76 ± 0.56	0.384	0.74 ± 0.58	0.54 ± 0.52	0.144

UCr: urine creatinine; Cr: creatinine; eGFR: estimated glomerular filtration rate; MMP-9: matrix metalloproteinase-9.

**Table 4:** Correlation analysis of urinary matrix metalloproteinase-9 and nephrin with selected renal parameters in idiopathic membranous nephropathy.

Renal parameters in IMN	Urinary nephrin (ng/*μ*mol Cr)		Urinary MMP-9 (ng/*μ*mol Cr)	
	*r*	*P* value	*r*	*P* value
Proteinuria (mg/*μ*molUCr)	0.174	0.073	0.332	0.015^∗^
eGFR (ml/min/1.73 m^2^)	-0.193	0.030^∗^	-0.279	0.025^∗^

IMN: idiopathic membranous nephropathy; eGFR: estimated glomerular filtration rate; UCr: urine creatinine; Cr: creatinine; MMP-9; matrix metalloproteinase-9; ∗: significant correlation.

## Data Availability

We did not obtain consent to share data in public. However, the data used in the current study will be availed to individuals by the corresponding author upon a reasonable request.

## Abbreviations

CKD: Chronic kidney disease
CKD-EPI: Chronic kidney disease epidemiology collaboration
CR: Creatinine
eGFR: Estimated glomerular filtration rate
ELISA: Enzyme-linked immunosorbent assay
ESRD: End-stage renal disease
IMN: Idiopathic membranous nephropathy
PLA_2_R: Phospholipase A_2_ receptor
TGF-*β*: Transforming growth factor-*β*
THSD7A: Thrombospondin type 1 domain-containing 7A.
